The article "Effect of Big Data Analysis-Based Remote Management Combined with Yangyin Runfei Decoction on Coagulation Function, Pulmonary Function, and Quality of Life of Pulmonary Tuberculosis Patients" was retracted in 2023. Reason: concerns about the peer review.

# Effect of Big Data Analysis-Based Remote Management Combined with Yangyin Runfei Decoction on Coagulation Function, Pulmonary Function, and Quality of Life of Pulmonary Tuberculosis Patients

**DOI:** 10.1155/2022/1708133

**Published:** 2022-04-25

**Authors:** Haihao Jin

**Affiliations:** Department of Traditional Chinese Medicine, The Third People's Hospital of Zhenjiang, Zhenjiang 212021, Jiangsu, China

## Abstract

**Objective:**

To explore the effect of big data analysis-based remote management combined with Yangyin Runfei decoction on coagulation function, pulmonary function, and quality of life (QOL) of pulmonary tuberculosis (PTB) patients.

**Methods:**

A total of 90 PTB patients treated in our hospital from May 2019 to May 2020 were selected as the subjects and divided into the experimental group (EG) and control group (CG) according to their admission order, with 45 cases each. Patients in CG accepted routine management and treatments and those in EG received big data analysis-based remote management combined with Yangyin Runfei decoction, so as to compare the clinical indicators between the two groups.

**Results:**

Compared with CG after treatment, EG presented an obviously higher total clinical effective rate, various pulmonary function indicators, and GQOLI-74 score (*P* < 0.001) and significantly lower various coagulation indicators and inflammatory factor indicators (*P* < 0.001).

**Conclusion:**

Performing big data analysis-based remote management combined with Yangyin Runfei decoction to PTB patients can effectively improve their QOL and pulmonary function and present a higher application value compared to routine management and treatments. Further research will be conducive to establishing a better solution for patients. This trial is registered with Clinical Study Registration Number: https://clinicaltrials.gov/ct2/show/ChiCTR2200057257.

## 1. Introduction

As a common disease in respiratory medicine, pulmonary tuberculosis (PTB) is mainly a pulmonary infectious disease triggered by Mycobacterium tuberculosis [1]. Clinically, PTB is characterized by bloody sputum, fatigue, and low-grade afternoon fever, which can trigger complications such as tuberculous pulmonary cavity and caseous pneumonia if no effective treatment is performed promptly, seriously compromising the life safety and reducing the quality of life (QOL) of patients [2, 3]. In addition, infection of the lungs by Mycobacterium tuberculosis can cause PTB, and factors such as drug abuse, immunocompromise, and alcohol, as well as poor sanitation, the very young and elderly group, and other personal factors, can also increase the risk of developing PTB. Rai Deependra et al. [4] stated that PTB has become one of the top ten lethal causes worldwide and that there are still millions of people suffering from PTB every year. The 5^th^ tuberculosis epidemiological random sampling survey in China reported that among the population aged over 15 years, about 4.95 million had active PTB, and the prevalence rate increased with the age, which reached the peak in people aged 74–79 years (about 1,539/100,000), and in different ages, the prevalence was always higher in men than in women [5, 6]. Motaharesadat et al. [7] stated that there were approximately 1.25 million deaths due to tuberculosis (TB) in 2017 worldwide. In addition, the Global Tuberculosis Report (2019) released by the World Health Organization (WHO) showed that there were still 9.98 million new TB cases in 2018 worldwide, mostly in the Southeast Asia region (42%), China remained one of the 30 countries with high TB burden, and the number of new TB patients in China each year was second only to India [8, 9].

The article "Effect of Big Data Analysis-Based Remote Management Combined with Yangyin Runfei Decoction on Coagulation Function, Pulmonary Function, and Quality of Life of Pulmonary Tuberculosis Patients" was retracted in 2023. Reason: concerns about the peer review.

PTB is featured by recurrent attack and long disease duration. At present, clinical treatment is mainly based on drug therapy, but it has a long treatment cycle, and persistent drug use can lead to obvious drug resistance and adverse effects, which, combined with poor medication adherence of patients, cause difficulty in achieving therapeutic effects. Some studies have pointed out that applying remote management based on big data analysis in modern drug therapy can improve clinical efficacy and prognosis [10]. Although conventional management and treatment modalities have a certain therapeutic effect, they are less effective in improving symptoms and recovering lung function. In addition, the conventional treatment fails to obtain the expected efficacy, and the conventional management cannot meet the clinical demands, and therefore, a new treatment modality is needed to improve the prognosis of PTB patients. Currently, the therapeutic effects of Yangyin Runfei decoction have been demonstrated in elderly patients with chronic obstructive pulmonary emphysema [11]. And Sudfeld et al. [12] confirmed that remote management based on big data analysis could improve maternal and infant outcomes and promote QOL of patients with gestational diabetes. But the combination of the two has rarely been reported. Based on this, combining big data analysis-based remote management with Yangyin Runfei decoction was adopted herein to carry out joint clinical intervention to the subjects, in the hope of providing a more clinical evidence-based basis for such patients.

## 2. Materials and Methods

### 2.1. General Data

A total of 90 PTB patients treated in our hospital from May 2019 to May 2020 were selected as the subjects and divided into the experimental group (EG) and control group (CG) according to their admission order, with 45 cases each. The study met the World Medical Association Declaration of Helsinki (2013) [13].

The article "Effect of Big Data Analysis-Based Remote Management Combined with Yangyin Runfei Decoction on Coagulation Function, Pulmonary Function, and Quality of Life of Pulmonary Tuberculosis Patients" was retracted in 2023. Reason: concerns about the peer review.

### 2.2. Enrollment of Study Subjects

Inclusion criteria were as follows: (1) patients who met the diagnostic criteria for PTB in the *National Health Commission of the People's Republic of China (WS 288-2017) Diagnosis for Pulmonary Tuberculosis Standards* [14], with the clinical manifestations including cough, night sweating, and hemoptysis; (2) patients who received chest imaging examination and presented acid-fast staining smear positive and TB sputum culture positive; (3) patients who obtained a positive result in the GeneXpert MTB/RIF test or presented typically pathologic tubercular changes; (4) patients who had normal language function and nerve function and could go along with the trial; (5) patients whose clinical data were complete; and (6) the study subjects who were long-term residents and could guarantee to complete the whole study period.

Exclusion criteria were as follows: (1) patients who had taken immunosuppressant or accepted relevant treatment before admission; (2) patients who had severe drug dependence; (3) patients who were pregnant or lactating women; (4) patients who were complicated with hematological disease and immune diseases; (5) patients who were complicated with other infectious diseases; (6) patients who had tumor; and (7) patients who participated in other trails.

### 2.3. Methods

#### 2.3.1. CG

*(1) Routine Management*. A management team was formed by the experienced chief physicians, attending physicians, and nursing personnel selected from the department of respiratory medicine to give one-to-one lessons to patients every 15 days, that is, informing the patients of the pathogenic factors, treatment key points, precautions, dietary intervention, medication instruction, health care, and other knowledge about PTB to relieve the patients' internal anxiety and depression and improve their treatment compliance; in addition, disinfection and isolation measures were strictly implemented, the wards were disinfected regularly, the patients were advised repeatedly to have enough rest and avoid overfatigue, and their condition was under real-time monitoring, so that any abnormalities could be taken care of by the physicians.

*(2) Drug Treatment*. The patients were administered with 0.1 g of levofloxacin tablets (manufacturer: Daiichi Sankyo Pharmaceutical (Beijing) Co., Ltd.; NMPA approval no. H20040091; specification: 0.5 g) once, three times a day for continuously 6 months.

The article "Effect of Big Data Analysis-Based Remote Management Combined with Yangyin Runfei Decoction on Coagulation Function, Pulmonary Function, and Quality of Life of Pulmonary Tuberculosis Patients" was retracted in 2023. Reason: concerns about the peer review.

#### 2.3.2. EG

*(1) Remote Management Based on Big Data Analysis*. Big data analysis-based remote management is a novel management method to perform remote monitoring diagnosis technology and deep learning-based remote intelligence-assisted diagnosis and treatment on the basis of routine management. The specific measures were as follows: (1) a management team was set up, which included nursing personnel with remote management experience, stronger communication ability, and professional knowledge of PTB remote management nursing. The team members received targeted training, mainly including the introduction of core idea of remote management based on big data analysis; (2) the management team members should timely establish the records for PTB patients, carry out telephone follow-up twice a week, regularly organize health education activities (once every 25 days), and provide support for the nursing demand of remote management, such as collecting health big data, integrating the trend prediction characteristics of heterogeneity, multiple sources, and collectiveness of big data with the homogeneous trace attribute of evidence-based medicine, learning the features of big data, extracting the core knowledge, and establishing the disease prediction model; (3) patients' condition changes were under real-time monitoring for increased sputum volume, aggravated symptoms of cough, fever, and hemoptysis, and the volume, rate, nature, and color of blood with the cough, and the occurrence of complications in patients was recorded timely; (4) patients' vital sign data were collected daily and uploaded in time to dig and predict the health status of each patient and perform multiangle analysis; (5) a TB healthcare knowledge map was constructed, and the dietary plan and exercise guidance were developed based on the actual situation of the patient and combined with data on patient health; (6) for the patients already admitted to the hospital, prompt treatment was given, and a differentiated intelligent diagnosis and treatment program was provided for the validation of remote intelligence-assisted diagnosis.

*(2) Yangyin Runfei Decoction*. The formula was 8 g of liquorice root, 11 g of prepared rehmannia root, 11 g of cochinchinese asparagus root, 11 g of stemona root, 11 g of Chinese angelica, 11 g of Chinese peony, 11 g of tendrilleaf fritillary bulb, 15 g of platycodon root, 15 g of dwarf lilyturf tuber, and 20 g of lily bulb. All herbs were decocted with water to 100 mL, and the decoction was taken in the morning and at night every day when it was still warm. The treatment lasted for 6 consecutive months.

### 2.4. Observation Indicators

The clinical efficacy was compared between the two groups. According to the CT scan, if the focus was absorbed completely, and the symptoms such as night sweating, hemoptysis, and cough disappeared, it was considered as cured; if most of the focus was absorbed, and the symptoms such as night sweating, hemoptysis and cough disappeared, it was considered as markedly effective; if the focus was absorbed to a certain extent, the volume of blood with the cough decreased, and the cough symptom was alleviated, it was considered as effective, and if the above vital signs and symptoms were not changed or were aggravated, it was considered as ineffective. The total clinical effective rate = (cured cases + markedly effective cases + effective cases)/total number of cases ∗ 100%.

The article "Effect of Big Data Analysis-Based Remote Management Combined with Yangyin Runfei Decoction on Coagulation Function, Pulmonary Function, and Quality of Life of Pulmonary Tuberculosis Patients" was retracted in 2023. Reason: concerns about the peer review.

After treatment, 5 ml of fasting venous blood was drawn from the patients in the two groups, the plasma was reserved after centrifugation, and the automatic coagulation analyzer (manufacturer: Jinan Yuxin Bio-tech Co., Ltd.; model: XL3200C) was used to test the coagulation indicators in all subjects, including thrombin time (TT), D-dimer level (D-D), fibrinogen (Fg), and platelet (PLT).

The pulmonary function detector (manufacturer: Hefei Jianqiao Medical Electronic Co., Ltd.; model: FGY-200) was used to test the pulmonary function indicators of patients in the two groups after treatment, including forced expiratory volume in one second (FEV_1_), the ratio of FEV_1_ over forced vital capacity (FVC) (FEV_1_/FVC), and peak expiratory flow (PEF).

5 ml of fasting elbow venous blood was drawn from all subjects in the morning, the serum was separated after centrifugation to extract the supernatant, all serum specimens were placed under -80°C, and the interleukin-6 (IL-6), procalcitonin (PCT), and tumor necrosis factor *α* (TNF-*α*) in the specimen were measured according to the specification of ELISA kits (manufacturer: Shanghai Fusheng Industrial Co., Ltd.).

The Generic Quality of Life Inventory-74 (GQOLI-74) [15] was used to evaluate the quality of life (QOL) of patients in the two groups after treatment. The scale contained 4 scoring items, that is, psychological functioning (mental strain, negative emotion, positive emotion, cognitive function, self-esteem), physical functioning (sleep and vigor, physical discomfort, eating function, sexual function, exercise, and sensation function), social functioning (social support, interpersonal skill, work and study, leisure life and entertainment, marriage and family), and material living conditions (housing, social service, living environment, economic status). The total score was 100 points, with higher scores indicating better QOL.

### 2.5. Statistical Processing

In this study, the data processing software was SPSS20.0, the picture drawing software was GraphPad Prism 7 (GraphPad Software, San Diego, USA), the items included were enumeration data and measurement data, the methods used were *X*^2^ test, *t*-test, and normality test, and differences were considered statistically significant at *P* < 0.05.

The article "Effect of Big Data Analysis-Based Remote Management Combined with Yangyin Runfei Decoction on Coagulation Function, Pulmonary Function, and Quality of Life of Pulmonary Tuberculosis Patients" was retracted in 2023. Reason: concerns about the peer review.

## 3. Results

### 3.1. Baseline Data

Table 1 shows that no significant between-group differences in gender, age, BMI value, course of disease, PTB type, educational degree, religious faith, and family income were observed (*P* > 0.05).

### 3.2. Clinical Efficacy

Table 2 shows that the total clinical effective rate was obviously higher in EG than in CG (*P* < 0.001).

### 3.3. Coagulation Indicators

Table 3 shows that various coagulation indicators were obviously lower in EG than in CG (*P* < 0.001).

### 3.4. Pulmonary Function Indicators

Table 4 shows that various pulmonary function indicators after treatment were obviously higher in EG than in CG (*P* < 0.001).

### 3.5. Inflammatory Factor Indicators

Table 5 shows that various inflammatory factor indicators after treatment were obviously lower in EG than in CG (*P* < 0.001).

### 3.6. GQOLI-74 Scores

Figure 1 shows that the GQOLI-74 score after treatment was obviously higher in EG than in CG (*P* < 0.001).

## 4. Discussion

Previous studies have shown that PTB mostly occurs in population with low body immunity, and those with crowded residence, poor life, and malnutrition are also susceptible to infection [16]. The disease mainly causes inflammatory damage in the lungs, which leads to respiratory dysfunction and seriously endangers the life and health of patients [17]. At present, early diagnosis and treatment are the main method for clinically treating PTB, so how to recognize PTB early and then carry out treatment is crucial for the prognosis of patients. Current conventional management is difficult to meet the needs of patients and is less detailed because the nursing measures were performed to patients within the given scope, so in clinical treatment it leads to poor patient treatment compliance and undesirable treatment effect [18]. By collecting big data, analyzing results, and summarizing the core, the remote management based on big data analysis can effectively inhibit the aggravation of the disease by means of carrying out targeted nursing work and diagnosis and treatment measures to the PTB patients and performing health education for patients to master disease-related knowledge and understand their condition changes anytime [19]. It was found in a study of 80 PTB patients conducted by Wahedi Katharina [20] that the remote management based on big data analysis could effectively improve patients' self-care ability and QOL, presenting significant promotion effect on prognosis and treatment effect. The manifestations of PTB symptoms are classified into the category of “lung consumption” in traditional Chinese medicine (TCM), and the theory of TCM considers deficiency of qi and blood and loss of yin and essence as the main factors triggering PTB [21]. Failed transpiration of body fluid due to lung deficiency causes the kidney losing the nourishment source and then leads to deficiency of kidney yin, unrecovered weakness, and deficiency of vital qi, resulting in MTB invading the lungs and compromised lung yin. Therefore, TCM holds that the treatment of PTB should be based on nourishment of yin, relieving cough, and eliminating phlegm [22]. The combination of multiple herbs in the Yangyin Runfei decoction has the effects of clearing deficient heat, clearing heat and cooling blood, invigorating yin and promoting fluid production, moistening lung for arresting cough, and nourishing essence and blood, so the decoction can effectively regulate viscera function and improve patients' clinical symptoms. Among these herbs in the Yangyin Runfei decoction, liquorice root has the effects of clearing heat and removing toxicity as well as relieving cough and reducing sputum, prepared rehmannia root can nourish blood and yin, cochinchinese asparagus root plays the role of nourishing yin for promoting fluid production and moistening dryness, etc., and platycodon root is able to ventilate lung qi for dissipating phlegm and relieve sore throat and expel pus. These herbs exert their effects together to alleviate the disease of patients. In this study, the total clinical effective rate was obviously higher in EG than in CG (*P* < 0.001), demonstrating that big data analysis-based remote management combined with Yangyin Runfei decoction could effectively improve clinical efficacy and promote rapid recovery.

The article "Effect of Big Data Analysis-Based Remote Management Combined with Yangyin Runfei Decoction on Coagulation Function, Pulmonary Function, and Quality of Life of Pulmonary Tuberculosis Patients" was retracted in 2023. Reason: concerns about the peer review.

The elevated D-D and Fg indexes represent that patients' body is in a hypercoagulable state, and they will further elevate with the aggravation of the disease. D-D has higher antigenicity, which is the product of fibrin after being hydrolyzed by plasmin, and its elevated level represents that patients' body fibrinolytic system is activated, and their blood is in a hypercoagulable state. A prolonged TT indicates an abnormality in the common coagulation pathway, and elevated PLT means a hyperfunctional state of the patient body, and the reason may be that tuberculosis bacteria lead to coagulation and thrombus and eventually trigger histopathological damage and cell adhesion [23, 24]. In this experiment, various coagulation indicators were obviously lower in EG than in CG (*P* < 0.001), indicating that big data analysis-based remote management combined with Yangyin Runfei decoction could effectively relieve the hypercoagulable state in patients' blood and achieve better treatment effect. In addition, with big data analysis, physicians can understand the vital signs of PTB patients and constantly adjust the nursing direction and measures, and the introduction of treatment measures on this basis can effectively improve the pulmonary function of patients. Cai et al. [25] stated that the body immune function of the patients can be impaired to various degrees during the progression of PTB, which stimulates the occurrence of inflammatory response, thereby further aggravating the condition. PCT is involved in the occurrence and progression of PTB, and the elevated PCT creates an imbalance in the anti-inflammatory-proinflammatory system of the body, which aggravates the inflammatory response and worsens the condition. In this study, after 6 months of treatment, various inflammatory factor indicators were obviously lower in EG than in CG (*P* < 0.001), implying that big data analysis-based remote management combined with Yangyin Renfei decoction could obviously lower the inflammatory factor expression and reduce the inflammatory reaction in the body. In addition, combining the multiple herbs in Yangyin Runfei decoction can eliminate oxygen-derived free radicals, resist oxidation, and enhance immune function in the body; meanwhile, this treatment modality also has immunomodulatory and anti-inflammatory effects, which can help to reduce inflammatory response in the body and improve immune function. By statistically analyzing the GQOLI-74 scale of the two groups, it was found that the GQOLI-74 score was obviously higher in EG than in CG (*P* < 0.001), demonstrating that combining big data analysis-based remote management with Yangyin Runfei decoction was positive in treating PTB and conducive to improving QOL, which was consistent with the current clinical study results. Shortcomings of the study: first, the cases selected in this study were patients treated in the local hospital, so the source and region of cases lacked diversity; second, limited by the observation time, the samples included in this clinical study were insufficient, leading to bias in the results; finally, scales were still the evaluation method in the clinic, so there would be certain subjectivity and intention when patients were answering the questions, which would affect the final results of the clinical trial to a certain extent. Moreover, patients from other provinces and nationalities were not included in the study, so the results may be affected by regional culture and ethnic difference. Therefore, study design should be improved in the future, with expanded sample size, perfected grouping, strict blind control, and objective evaluation of cognitive function indicators, etc., so as to obtain more rigorous and objective data and conclusion.

The article "Effect of Big Data Analysis-Based Remote Management Combined with Yangyin Runfei Decoction on Coagulation Function, Pulmonary Function, and Quality of Life of Pulmonary Tuberculosis Patients" was retracted in 2023. Reason: concerns about the peer review.

## Figures and Tables

**Figure 1:** Between-group comparison of GQOLI-74 scores ($\bar{x}\pm s$). Note: the horizontal axis indicated EG and CG, and the vertical axis indicated the GQOLI-74 score (points), the GQOLI-74 scores of EG and CG were, respectively, (76.02 ± 3.27) and (55.60 ± 3.19), and ^*∗*^indicated a significant between-group difference in GQOLI-74 scores after treatment (*t* = 29.985, *P* < 0.001).

**Table 1:** Between-group comparison of baseline data.

Item	EG (*n* = 45)	CG (*n* = 45)	*x* ^2^/*t*	*P*
Gender			0.049	0.824
Male	29 (64.44%)	30 (66.67%)		
Female	16 (35.56%)	15 (33.33%)		
Age ($\bar{x}\pm s$, years)	49.91 ± 13.16	48.76 ± 12.63	0.423	0.673
BMI (kg/m^2^)	20.65 ± 0.88	20.50 ± 0.85	0.822	0.413
Course of disease ($\bar{x}\pm s$, years)	3.87 ± 1.34	3.29 ± 1.12	0.228	0.028
PTB type				
Infiltrative	15 (33.33%)	16 (35.56%)	0.049	0.824
Primary	13 (28.89%)	14 (31.11%)	0.053	0.818
Disseminated	9 (20.00%)	8 (17.78%)	0.073	0.673
With chronic fibrous cavity	8 (17.78%)	7 (15.56%)	0.080	0.777
Educational degree				
Primary school and junior high school	16 (35.56%)	17 (37.78%)	0.048	0.827
Senior high school and junior college	13 (28.89%)	14 (31.11%)	0.053	0.818
College and above	16 (35.56%)	14 (31.11%)	0.200	0.655
Religious faith			0.049	0.824
Yes	15 (33.33%)	16 (35.56%)		
No	30 (66.67%)	29 (64.44%)		
Family income			0.047	0.829
≥3,000 yuan (month·person)	27 (60.00%)	28 (62.22%)		
<3,000 yuan (month·person)	18 (40.00%)	17 (37.78%)		
Place of residence			0.045	0.832
Urban area	26 (57.78%)	25 (55.56%)		
Rural area	19 (42.22%)	20 (44.44%)		

**Table 2:** Between-group comparison of clinical efficacy (*n*(%)).

Group	*N*	Cured	Markedly effective	Effective	Ineffective	Total clinical effective rate
EG	45	8 (17.78%)	13 (28.89%)	20 (44.44%)	4 (8.89%)	41 (91.11%)
CG	45	3 (6.67%)	9 (20.00%)	14 (31.11%)	19 (42.22%)	26 (57.78%)
*x* ^2^						13.141
*P*						<0.001

**Table 3:** Between-group comparison of coagulation indicators ($\bar{x}\pm s$).

Group	*N*	TT (s)	D-D (mg/L)	Fg (g/L)	PLT (^*∗*^10^9^/L)
EG	45	16.03 ± 0.89	0.38 ± 0.04	2.06 ± 0.15	200.74 ± 10.58
CG	45	20.38 ± 1.00	0.81 ± 0.14	3.52 ± 0.24	236.28 ± 12.68
*t*		21.798	19.811	34.605	14.437
*P*		<0.001	<0.001	<0.001	<0.001

**Table 4:** Between-group comparison of pulmonary function indicators ($\bar{x}\pm s$).

Group	*N*	FEV_1_ (L)	FEV_1_/FVC (%)	PEF (L/min)
EG	45	2.53 ± 0.26	76.55 ± 3.51	397.78 ± 28.43
CG	45	1.78 ± 0.25	68.93 ± 2.77	357.92 ± 31.91
*t*		13.949	11.432	6.257
*P*		<0.001	<0.001	<0.001

The article "Effect of Big Data Analysis-Based Remote Management Combined with Yangyin Runfei Decoction on Coagulation Function, Pulmonary Function, and Quality of Life of Pulmonary Tuberculosis Patients" was retracted in 2023. Reason: concerns about the peer review.

**Table 5:** Between-group comparison of inflammatory factor indicators ($\bar{x}\pm s$).

Group	*N*	IL-6 (g/L)	PCT (ng/mL)	TNF-*α* (g/L)
EG	45	9.18 ± 1.65	0.14 ± 0.01	9.05 ± 1.23
CG	45	16.34 ± 3.69	0.42 ± 0.03	17.41 ± 1.77
*t*		11.883	59.397	26.019
*P*		<0.001	<0.001	<0.001

## Data Availability

The data used to support the findings of this study are available on reasonable request from the corresponding author.
